The article "Mutation Detection and Functional Analysis of MSX1, PAX9, AXIN2, and BMP in Nonsyndromic Congenital Missing Teeth Based on Intelligent Image Detection" was retracted in 2023. Reasons: signs of a paper mill; suspected computer-generated content; unreliable results or conclusions; concerns about the data.

# Mutation Detection and Functional Analysis of MSX1, PAX9, AXIN2, and BMP in Nonsyndromic Congenital Missing Teeth Based on Intelligent Image Detection

**DOI:** 10.1155/2022/6217399

**Published:** 2022-05-20

**Authors:** Xueqin Yao, Cheng Zhang, Peipei Gao, Zixuan Meng, Yonghong Hao, Jingjing Yan, Wenbo Yao

**Affiliations:** Pediatric Stomatology of Beijing Tongzhou Xinhua Hospital, China

## Abstract

Due to the complexity of clinical manifestations and the lack of standardized diagnostic criteria, it is still difficult to distinguish the etiological types of congenital edentulousness corresponding to genetic defects. This paper studies the application of deep learning image processing and digital image processing in medical images in detail and analyzes the functions of congenital edentulous hotspot genes. The cases in the control group and the study group were collected, and the gene mutations of direct sequence MSX1, PAX9, AXIN2, and BMP were analyzed, and new pathogens were found. The experimental results suggest that PAX9 and MSX1 genes may have a synergistic effect in nonsyndromic congenital edentulous patients. In severely missing teeth, the role of PAX9 may be greater than that of MSX1. The experimental results will help us lay the foundation for further understanding of the disease in the future.

## 1. Introduction

Congenital tooth loss is a disease of dental hypoplasia that only manifests as the loss or abnormality of the number of teeth, which belongs to the number hypoplasia in congenital dental hypoplasia [1, 2]. Congenital lack of teeth affects the normal development of the oral and maxillofacial system of patients, causing developmental deformities of the craniomaxillofacial region, which further affects the patient's appearance (such as bony crossbite and midface collapse), pronunciation, facial aesthetics, general development, and mental health. These complications are seriously endangering people's physical and mental health. In addition, congenitally missing teeth are often accompanied by allergic diseases [3, 4].

The clinical manifestations of nonsyndromic congenital edentulous generally involve the permanent dentition, rarely involving the deciduous dentition, the third molar is most often missing, and the number of other teeth is variable. There are obvious racial differences in missing teeth. Except for the third molars, the most common missing teeth in Asian populations are mandibular incisors, and the most common ones in European and American populations are mandibular second premolars and maxillary lateral incisors. After tooth loss, the chewing efficiency is reduced or even lost, which increases the burden on the gastrointestinal system, reduces the quality of life, and affects aesthetics and mental health.

Using computer technology to extract the basic information of teeth in panoramic X-ray films can significantly reduce the workload of doctors [5]. Weon et al. have developed an algorithm for fusing a 3D LIDAR (Light Detection and Ranging) system that receives objects detected in a deep learning-based image sensor and object data in the form of 3D point clouds. Match 3D LIDAR data to 2D image data through fusion of mixed-level multisensors. First, since 3D LIDAR data represents all objects within the sensor's detection range as points, all unnecessary data, including ground data, is filtered out. The 3D Random Sample Consensus (RANSAC) algorithm can extract ground data perpendicular to the reference estimated 3D plane and data at both ends through ground estimation [6]. Divya and Leena utilize smart devices for fall detection. Vision-based detection with compressed neural networks running on smart devices built using transfer learning. Leverage image augmentation to build datasets to improve model performance. The model is evaluated in terms of accuracy, and the strength of the fog layer is evaluated in terms of latency. Compared with the existing state-of-the-art algorithms available for detection, the accuracy of the proposed model is 98.5% [7]. It is of practical significance to study the mutation detection of congenital missing teeth by intelligent image detection.

At present, the epidemiological investigation and genetic research on congenitally missing teeth in my country is basically blank. In view of this situation, in order to explore the mutation detection in nonsyndromic congenitally missing teeth, this paper carried out the incidence of such diseases in the population and analyzed them. It was found that the mutation detection of the disease was different in MSX1, PAX9, AXIN2, and BMP, and there were statistically significant differences. In conclusion, the study of the clinical characteristics and pathogenesis of congenital edentulous patients not only has a clinical diagnosis and treatment of the disease. It has important guiding significance and also has important practical significance for the etiology research of the disease.

## 2. Mutation Detection and Functional Study in Nonsyndromic Congenital Edentulous

### 2.1. Deep Learning Image Processing

Deep convolutional neural networks enable complex training models of traditional machine learning algorithms [7]. The structure of the convolutional neural network is shown in Figure 1. It has a fixed-size convolution kernel and an input image that performs integration to capture features such as edges, textures, and contours in the image. The pooling layer is also based on a fixed size. The scale is downsampling, so that the receptive field of the feature image can be enlarged according to the scale [8, 9]. Then, the obtained feature information is mapped to a fixed-length feature vector through the fully connected layer to achieve the effect of classification.

In practical applications, the scale of medical image databases is always small, and in the eyes of complex models, training from scratch can easily lead to overcorrection. To avoid this, preliminary descriptions of models have become a common practice. This feature directly uses some template templates on ImageNet and COCO datasets [10]. In this case, the pre-existing templates act as feature suppliers, and they can restore the data simply by replacing the new layers in the new template [11].

### 2.2. Digital Image Processing

Image augmentation is often employed when faced with small sample image datasets. Since most medical image datasets are small sample datasets, these techniques are often used in the image enhancement process of medical images [12].

Commonly used basic image enhancement methods include cropping, flipping, rotating, adding noise, filtering, and sharpening [13]. Taking horizontal mirroring as an example, if the height and width of an image are known as (*l*Height, *l*Width), set the coordinates of a point in the image to be (*x*0, *y*0), and after horizontal mirroring, the coordinates of this point will become (*l*Width − *x*0, *y*0), which can be expressed as follows:

(1) $$\begin{array}{c} \left[\begin{array}{c} x1\\ y1\\ 1 \end{array}\right]=\left[\begin{array}{ccc} -1 & 0 & l\text{width}\\ 0 & 1 & 0\\ 0 & 0 & 1 \end{array}\right]\left[\begin{array}{c} x0\\ y0\\ 1 \end{array}\right]. \end{array}$$

The inverse operation matrix expression is as follows:

(2) $$\begin{array}{c} \left[\begin{array}{c} x0\\ y0\\ 1 \end{array}\right]=\left[\begin{array}{ccc} -1 & 0 & l\text{width}\\ 0 & 1 & 0\\ 0 & 0 & 1 \end{array}\right]\left[\begin{array}{c} x1\\ y1\\ 1 \end{array}\right]. \end{array}$$

To realize the mirror image of the whole image, all the points in the image need to be calculated. Similarly, the realization of vertical mirroring is to change the coordinates of all points (*x*0, *y*0) to (*x*0, *l*Height − *y*0) [14].

The noise in the image can be regarded as the interference signal in the image signal. For example, “snowflakes” in a TV image can be seen as image noise that interferes with the original image. In the process of image acquisition, various problems such as equipment and environment often cause interference and introduce image noise, thereby affecting the image quality [15]. Therefore, in the process of image enhancement, filtering is usually used to remove noise. In data enhancement, in order to increase the diversity of the data, noise will be artificially added to the image.

The main purpose of image sharpening is to make blurry images clear. Image sharpening methods are usually divided into two types: one is the differential method, which mainly enhances the pixels with large gradients through image gradient operations to highlight image details, so as to achieve the purpose of sharpening. The other is to use high-pass filtering to accept high-frequency signals and suppress low-frequency signals, thereby highlighting the details of the image and sharpening the image [16]. Both methods are now more popular image sharpening methods.

### 2.3. Dental X-Ray Images

In dentistry, X-ray examinations are divided into two categories: intraoral X-ray examination, which is a technique in which a film is placed in the mouth, that is, the X-ray image is obtained in the patient's mouth, and a technique placed between the radiograph and the X-ray source, where the X-ray image is acquired outside the patient's mouth. This results in the following types of X-ray images: bitewing, apical (intraoral), and panoramic (extraoral) [17].

The bite wing X-ray image is used to display the details of the upper and lower teeth in the oral area, while the periapical X-ray image is used to monitor the entire tooth, which can display the enamel, dentin, cementum and other dental hard tissues and pulp soft tissues [18]. Panoramic radiography, also known as orthodontic radiography, is a radiological examination that can obtain basic information for the diagnosis of dental abnormalities.

### 2.4. Congenital Missing Tooth Hotspot Genes

#### 2.4.1. PAX9

The PAX transcriptional gene family plays an integral role in vertebrate ontogeny [19]. All members of this family have a paired control domain, an octapeptide domain, and a paired homology domain. These structures play an important role in fetal development and tumor formation. As a transcription factor, it has the ability to bind to DNA. PAX9 is involved in a variety of regulatory mechanisms and plays a crucial role in tumorigenesis. PAX9 is highly expressed in salivary gland tumors, especially malignant tumors, and may play a negative role in the prognosis of patients with esophageal squamous cell carcinoma [20]. Regular screening of patients with PAX9 gene mutations is essential for clinical screening, especially for tumors in tissues with high PAX9 expression such as esophagus, salivary glands, prostate, lung, thyroid, and bladder [21].

#### 2.4.2. MSX1

MshHomeobox1 (MSX1) is located on human chromosome 4 q.16.2 with a full length of 5.6 k bases, including two exons. As a negative regulator of tooth differentiation, it plays an important role in tooth differentiation and development. Abnormalities of this gene not only show abnormal number of teeth but also affect the morphological development of teeth. Mutations in this gene are highly associated with congenital edentulous and nonsyndromic cleft lip and palate in humans. The MSX1 gene exhibits cleft lip, cleft palate, and dental developmental disorders and affects development. The effect of MSX gene mutation seems to be caused by its influence on downstream genes. The lack of MSX1 gene downregulates the expression of downstream gene BMP4 and transcription factor LEF. Through a series of complex biological regulation, it leads to tooth loss and the formation of cleft lip and palate.

#### 2.4.3. AXIN2

AXIN2 is a central axis arrestin 2 gene, located on chromosome 17 q.23, with a full-length gene of 43 k bases, including 10 exons. The transcribed mRNA is 4241 bases, the CDS translation transcript is 2532 bases, and the translation forms 843 amino acids. This gene encodes axon arrestin 2, which mainly functions as a structural support protein and plays an important role in the WNT signaling pathway. AXIN protein regulates the expression level of *β*-catenin in the nucleus by negative feedback and maintains the stability of *β*-catenin inside and outside the cell. In the absence of WNT pathway ligands, *β*-catenin can still stimulate the continuous action of the signaling pathway. The deficiency of *β*-catenin hinders the excitation of WNT signaling pathway and destroys the second important function of *β*-catenin-adhesion function.

#### 2.4.4. BMP signaling pathway

USAG-1 (uterine sensitization associated gene-1, uterine sensitivity-related gene) is a BMP antagonist and can regulate the WNT signaling pathway. Murashima-Suginami et al. found that USAG-1-deficient mice developed multiple teeth with enhanced BMP signaling. Subsequent studies found that blockade of BMP signaling could relieve the formation of supernumerary teeth.

The fine regulation of these signal molecules is very important to maintain the proper number of teeth, such as the inhibition of Shh signal expression in the early stage of tooth germ development and the regulation of WNT signal expression. Epiprofin is expressed in tooth germ epithelium and can interact with BMP, Shh, and WNT signaling pathways and participate in the regulation of the number of teeth. In mice lacking Epiprofin expression, supernumerary incisors and molars can be seen. In addition, inactivation of IL11 signaling can cause craniosynostosis, maxillary dysplasia, delayed tooth eruption, and the occurrence of supernumerary teeth.

## 3. Investigation and Study of Mutation Detection and Function in Nonsyndromic Congenital Absence of Teeth

### 3.1. Research Objects

The cases in the research group came from patients who were treated in the Dental Clinic Center of Xinhua Hospital in Tongzhou District. After excluding the history of tooth extraction, X-ray examination confirmed that there was no permanent tooth germ in the edentulous area. The number of simple missing teeth (except third molars) with no syndrome and more than 10 teeth was selected. Congenital edentulous patients or other developmental deformities were included in the study group after informed consent. The frequency of tooth loss in each tooth position of the 10 patients is shown in Figure 2.

*Control group case selection*: 100 noncongenitally edentulous patients were randomly selected as normal controls, 50 males and females, aged between 20 and 60 years old, screened the found mutations of unknown pathogenic nature, and further excluded the mutation as possibility of SNP. If the mutation does not exist in the normal population, it suggests that it is a possible pathogenic mutation; if the mutation exists in the normal population, it suggests that it may be a SNP.

### 3.2. Experimental Reagents

1. *Red blood cell lysate*: provided by the Laboratory of Molecular Biology Technology, Medical University
2. *Isopropyl alcohol and anhydrous ethanol*: all of analytical grade, products of Bengbu Chemical Reagent Factory
3. *Tris-phenol*: product of M company
4. *Chloroform*: analytically pure, chemical preparation factory product
5. *Proteinase K*: provided by the Laboratory of Molecular Biology Technology, Medical University

### 3.3. Experimental Method

1. Backup preservation of genomic DNA and preparation of template DNA

Measure the purity and concentration of the DNA stock solution using a spectrophotometer and divide it into 2-3 tubes. One is kept in a freezer at -80°C and the rest at -20°C and 4°C for DNA detection and analysis.

Prepare template DNA at a concentration of 50 ng/*μ*l depending on the concentration of the DNA stock.

(2) Gene primer design

The length of primers was controlled at 16~24 bp.

The GC content is controlled between 40% and 60%.

The primers themselves cannot have 4 consecutive bases complementary.

The energy values of primer dimers and hairpin structures should not be too high.

(3) Polyacrylamide gel electrophoresis

After amplification, take 2 *μ*l of PCR amplification product, use 6% polyacrylamide gel (30% acrylamide 6 ml, 10× TBE 1.5 ml, TEMED409l, and 10% APS30091, add distilled deionized water 30 ml) electrophoresis detection, 300 V constant pressure. Electrophoresis was performed for 50 minutes, stained with silver nitrate, and the results were observed and recorded.

## 4. Mutation Detection and Functional Analysis and Research in Nonsyndromic Congenital Missing Teeth

### 4.1. Sequencing Results of PAX9 Gene

In the sequencing results of the PAX9 gene, there is a heterozygous/homozygous mutation of c.631+41g>a in the intron position of 41 bases downstream of exon 1. After searching the SNP database, it was found that he was an intron SNP site (No. rs5214607), so the site is far away from the exon, and it does not participate in the coding of proteins and does not affect the splicing site at the end of the exon, so it is a nonpathogenic polymorphism.

There is a heterozygous or pure sum mutation of c.717-718CG>TC in exon 2 of PAX9 gene. There are 5 main sequencing results of these two loci, as shown in Table 1. The heterozygous change at position 717 causes the amino acid codon CAC to change to CAT, which is still a histidine codon, c. The heterozygous change at position 718 causes the amino acid codon GCG to change to CCG, and the amino acid changes from alanine to histidine. After searching the SNP database, it was found that these two loci are SNP loci, numbered rs6254140 and rs9251432, and the control test of a large sample of normal people proved that they were nonpathogenic mutations. However, by analyzing the results of this study, it can be found that it can be determined that the heterozygous double peak caused the structural change of the DNA template strand, which showed double bands in electrophoresis; The cases with heterozygous mutation, that is, heterozygous double peaks, occupy a certain proportion of 3/10, and the proportion is relatively large. It can be speculated that it has an impact on the pathogenic factors of congenital edentulous.

### 4.2. Sequencing Results of MSX1 Gene

In the sequencing results of MSX1 gene, the detected SNP loci are as follows: C.119C>G pure and change on exon 1, and after searching the SNP database, it is found that it is an exon SNP locus (number rs62514851). For exon 1 c.348C>T heterozygous/homozygous change, after searching the SNP database, it was found that it was an exon SNP site (number rs825146241). The above two sites have a large sample of normal people controlled studies abroad, indicating that the base changes at these two sites are not the cause of congenital lack of teeth directly, and we can speculate that it is an indirect cause of congenital lack of teeth. There is a t insertion change at the c.470.24 intron upstream of exon 2. After searching the SNP database, it is found that it is an exon SNP site (number rs5618512). Due to the insertion of a single base, a unidirectional repeat appears in the sequencing results. Sequence and electrophoresis result is a single band, indicating that the DNA structure has not changed, and this insertion mutation due to repeated base sequence is a common SNP site, which is a nonpathogenic polymorphic change. The heterozygous change of c>t in the intron position c.912+68 downstream of exon 2 was searched in the SNP database, and it was found that it was an exon SNP site (number rs6914), so the site was far away from the exon, and it was not participating in coding proteins does not affect the splice site at the end of the exon, so it can be determined to be a nonpathogenic polymorphic change.

The relationship between lineage genotype and edentulous interval can be found. In this study, most patients with missing teeth were concentrated in the anterior teeth area. When the posterior teeth were missing, PAX9 had a greater impact than MSX1. The relationship between genotype and the missing teeth interval is shown in Table 2.

PAX9 has 8 anterior teeth and 7 posterior teeth, as shown in Figure 3. In summary, the two genes PAX9 and MSX1 may have a synergistic effect in patients with simple congenital edentulousness.

### 4.3. Analysis of AXIN2 Sequencing Results

The sequencing results of this study showed that the codon corresponding to the 264th position of exon 2 changed from ACA→GCA, threonine to alanine, and a missense mutation occurred; the 547th position CAA→CGA, glutamine changed from arginine, and a missense mutation also occurred. At position 162 of exon 6, CCG→CTG, a missense mutation occurred, and proline was changed to leucine. At position 922 of exon 11, GAT→GAG, a missense mutation occurred, and the aspartic acid was changed to glutamic acid; the position 1141, ACT→ACA, still encoded threonine, and a synonymous mutation occurred. No mutation sites were found in DNA testing of 100 healthy controls.

### 4.4. Analysis of BMP Sequencing Results

The Ct value of the sample qRT-PCR detection results is shown in Table 3, and the amplification of PAX9 and BMP genes is shown in Figure 4.

In the overall analysis, the genotype distribution of only two BMP polymorphisms, rs2518516 and rs42815, was significantly different between cases and controls among the five loci (rs2518516, *P* = 0.028 and rs42815, *P* = 0.032), which is the first time that two loci associated with missing teeth were found in this study. In a stratified analysis by edentulous type, the recessive models of rs3178250 and rs15705 were associated with congenital loss of lower incisors and increased the risk of congenital loss of lower incisors compared with wild type (rs2518516, ORrec = 1.50 and rs42815, ORrec = 1.42). The recessive model and mutant homozygotes of rs235768 have a protective effect on congenital odontogenesis compared with the wild type.

## 5. Conclusions

Nonsyndromic congenital missing teeth are common in clinic. Most of the existing solutions are to restore the missing part through various clinical repair methods, but the effect is not ideal. If the disease can be completely prevented and intervened from the pathogenesis, it would be a major breakthrough. In this paper, the gene mutation detection in the research group and the control group collected through the investigation and combined with clinical analysis, the following conclusions are drawn: several popular genes PAX9, MSX1, EDA, AXIN2, etc. Missing teeth and related diseases (cleft lip and palate, ectodermal hypoplasia, colorectal tumorigenesis, etc.) have research significance. The heterozygosity change of PAX9 gene c.717.718CG>TC may be the cause of the disease in patients with simple congenital edentulous. MSX1 gene c.469+5G>A heterozygous mutation is a pathogenic mutation in severe nonsyndromic congenital edentulous. In addition, the homozygous change of c.119C>G and the heterozygous change of c.348C>T may also be the cause of the onset of nonsyndromic congenital edentulous patients.

## Figures and Tables

**Figure 1:** Typical convolutional neural network structure.

**Figure 2:** Frequency of tooth loss in each tooth position in 10 patients.

**Figure 3:** Relationship between genotype and edentulous interval.

**Figure 4:** PAX9 and BMP gene amplification Ct values.

**Table 1:** Classification of sequencing results at position c.717.718 of the PAX9 gene.

Cdna.717	Cdna.718	Electrophoresis results
Without	G>C pure	Single strip
G>C miscellaneous	Without	Single strip
Without	C>T pure	Single strip
C>T miscellaneous	Without	Single strip
C>T miscellaneous	G>C miscellaneous	Two belts

**Table 2:** Relationship between genotype and edentulous interval.

Genotype	Front teeth	Back teeth
MSX1 mutation	4	2
PAX9 mutation	8	7
Both genes have mutations	11	5
Without	1	1

**Table 3:** PAX9 and BMP gene amplification Ct values.

Sample	Ct duplicate 1	Ct duplicate 1	Ct duplicate 3	Internal reference Ct duplicate well 1	Internal reference Ct duplicate well 2	Internal reference Ct duplicate well 3
mut-PAX9	25.47	25.55	25.63	25.14	25.98	25.46
nor-PAX9	24.61	24.11	24.21	23.11	23.10	23.28
mut-BMP	28.14	28.06	28.30	24.88	24.79	24.92
nor-BMP	22.08	22.39	22.63	23.89	23.99	23.68

## Data Availability

The data underlying the results presented in the study are available within the manuscript.
